# New Auxiliary Function with Properties in Nonsmooth Global Optimization for Melanoma Skin Cancer Segmentation

**DOI:** 10.1155/2020/5345923

**Published:** 2020-04-13

**Authors:** Idris A. Masoud Abdulhamid, Ahmet Sahiner, Javad Rahebi

**Affiliations:** ^1^Department of Mathematics, Suleyman Demirel University, Isparta, Turkey; ^2^Department of Electrical and Computer Engineering, Altinbas University, Turkey

## Abstract

In this paper, an algorithm is introduced to solve the global optimization problem for melanoma skin cancer segmentation. The algorithm is based on the smoothing of an auxiliary function that is constructed using a known local minimizer and smoothed by utilising Bezier curves. This function achieves all filled function properties. The proposed optimization method is applied to find the threshold values in melanoma skin cancer images. The proposed algorithm is implemented on PH2, ISBI2016 challenge, and ISBI 2017 challenge datasets for melanoma segmentation. The results show that the proposed algorithm exhibits high accuracy, sensitivity, and specificity compared with other methods.

## 1. Introduction

Skin cancers are the most widely recognised type of growths in humans. They are a type of destructive disease that affects skin [1]. Most skin growths are reparable during the early stages. Therefore, the early diagnosis of skin tumours can save patients. Nowadays, computers and intelligent handheld devices are common and therefore can help diagnose melanoma earlier. Computer-Aided Diagnosis (CAD) tools can be connected to such devices to create a smart system that helps dermatologists recognize the melanoma. Moreover, Codella et al. [2] have shown in recent research that some of these CAD systems have better performance than average human expert agreements. Traditional melanoma detection CAD programs generally consist of three main components: the segmentation of the lesion, the extraction of functions, and the classification of features [3]. Yu et al. [4] showed that although melanoma patients can only be classified by means of features extracted using deep study models, the diagnostic performance is significantly improved by incorporating segmented lesions.

Numerous problems in the fields of engineering, economics, and natural sciences can be represented as global optimization problems. Thus, from a technical and scientific point of view, it is becoming increasingly important to study and develop methods that can solve this class of difficult mathematical problems. Currently, numerous new theoretical and practical methods have been reported to search for the global optimum. The one-dimensional optimization method is one of the most effective approaches for this purpose. This method is based on selecting directions randomly. The group of one-dimensional algorithms is referred to as line search methods [5]. They define an algorithm in which the direction of search is determined randomly at each iteration. This class of optimization methods is used as a part of descent techniques, which depend on objective function derivatives. The filled function method was produced by Ge (1990) [6]. It is produced with respect to passing from the current local minimizer to the lower one until the global minimizer is determined. Numerous classes of filled functions have been introduced by several authors (see, e.g., [6–12]). Bezier curves were introduced to solve the nonsmoothness of curves. They were developed by Pierre Bezier in 1962 for the styling of motorcar bodies [13]. Currently, Bezier curves are broadly used in computer graphics and animation. They are normally used for curve and surface design. In this study, a new auxiliary function with properties in nonsmooth global optimization is developed. This auxiliary function achieves all filled function properties, and it is used for finding the threshold value in melanoma skin cancer images. Even though the proposed algorithm has demonstrated powerful in both local and global searches and can be widely used in various optimization problems, it has some limitations including parameters adjustment, as it is a delicate task since it directly affects the efficiency of the auxiliary function. This paper contributes to the development of melanoma detection using new auxiliary function with properties in nonsmooth global optimization algorithm. In this study, the melanoma in the dermoscopic images was detected by three steps. The red channel on the colored dermoscopy image is selected in the preprocessing step. A 2*D* median-size 25∗25 filter and morphological filtering based on the Gaussian kernel have been used for smoothing. The following step was to determine the optimum melanoma segmentation threshold value using the proposed algorithm. Eventually, the estimated optimum threshold value has been used as the thresholding method used in the Otsu [14]. In order to demonstrate the effectiveness of this study, the proposed method has been evaluated on three public dermoscopic image databases: PH2 [15], ISBI2016 challenge [16], and ISBI 2017 challenge [17]. This paper is organized as follows. In Section 2, related works are viewed. In Section 3, the new method is presented, preceded by preliminaries and assumptions related to global optimization. In Section 4, the melanoma detection using global optimization algorithm is proposed. Evaluation results with comparisons are reported in Section 5. Finally, the conclusion of the study is remarked in Section 6.

## 2. Related Works

The conventional method for determining skin malignancy is the biopsy technique [3, 18]. In this technique, skin is scratched or evacuated, and samples are collected for research and testing. Computer-based skin disease location is beneficial to patients because patients can distinguish skin tumours without visiting a healing centre or without the assistance of a specialist [3].

Xie et al. [19] proposed novel convolutional neural network for skin lesion segmentation. In their method, they generated high-resolution feature maps to preserve spatial details. For the enhancement of features, the special and channel-wise mechanism was adopted.

Hwang and Celebi [20] solved surface in skin figures and applied mathematical approaches such as the gray stage coprevalence matrix. They reported that surface investigation may exactly detect the boundary with a smooth surface, and such surface study is the segmentation of dermatological images [21, 22]. Mishra and Celebi [23] reported the detection of skin abnormalities (particularly melanomas) using image processing methods and machine learning. Melanoma is typically considered as a dull-raised injury; these tumours develop from colored cells. A few melanomas lose color, having no or almost dull shade, and they can appear pink, white, or tan. Melanomas are considered to be the most dangerous of skin growths. Even though Merkel cell carcinoma is lethal in most cases, melanoma generally causes more deaths than several other types of skin disease. According to the American Cancer Society, approximately 76,380 (46,870 male and 29,510 female) new instances of melanoma were reported in 2016, among which 10,130 cases were fatalities (6750 male and 3380 female). The frequency of melanoma has been rising globally each year. Numerous lives can be saved if melanomas can be identified at the earliest stages when they are effectively treatable. Various examination methods based on different advances are being widely developed for the early identification of melanoma.

Jain and Pise [24] proposed methods of detecting melanoma skin cancer using computer systems and image processing. Numerous studies have demonstrated that computer vision can play a vital role in medical image diagnosis. The contribution to the framework was the skin sore figure. After that, by applying novel figure preparing procedures, it is examined to finish near the skin growth.

Jaleel et al. [25] detected skin cancer using computer systems. The biopsy technique is commonly used for skin disease recognition. In biopsy, skin is evacuated or scratched and samples undergo extensive testing. Computer-based skin growth identification is beneficial to patients who can distinguish a skin malignancy without visiting a healing centre or without the assistance of a specialist. Computer-based identification utilises imaging strategies and artificial intelligence. The distinctive phases of identification include the accumulation of dermoscopic figures, search of the figures for expelled hairs and noise, fragmentation of the figures by utilising the maximum entropy threshold, extraction of highlights using a gray level coevent matrix, and arrangement by employing an artificial neural network. A backpropagation neural network is utilised for ordering. It categorises a given informational index as cancerous or noncancerous.

Esteva et al. [26] proposed techniques for the segmentation of different types of skin carcinoma. Profound convolutional neural networks (CNNs) indicated the potential for general and specific factor assignments crosswise over multiple fine-grained protest classes.

Ramlakhan and Shang [27] proposed a classification system for cancerous skin lesions. In their technique, a model of a figure was constructed by a robotised melanoma acknowledgement framework using Android cell phones. The framework comprised of three noteworthy segments, i.e., figure division, computation, and characterisation. It was intended to be run on a cell phone with a camera or on a tablet computer. Hoshyar et al. [28] investigated the automated early detection of skin malignancy. Dermatology imaging researchers assumed that finding skin melanomas can be automated based on certain physical features and shading information that are typical of the characterisations of skin tumours. Goyal and Jain [29] reported the computer-based automated detection of melanoma skin malignancy. Melanoma skin tumours occur when shade-producing cells (melanocytes) grow uncontrollably, and these tumours result in pain.

Karargyris et al. [30] proposed a new application for image processing to identify skin malignancy using a smartphone. Xu et al. [31] proposed a technique for the analysis and classification of melanocytic skin cancer. The proposed technique contains four essential modules. In the first module, a multiassurance framework parcels the epidermis and dermis zones. Next, an epidermis examination is performed, in which the nuclear morphologies and spatial spreads of the epidermis features are investigated.

Li and Shen [32] proposed a method of analysing skin lesions using a deep learning network. Two deep learning techniques were proposed to address three principle aspects in the field of skin injury figure manipulation, i.e., sore division, sore dermoscopic highlight extraction, and sore characterisation. A deep learning system composed of two completely coevolutionary residual networks (FCRNs) is proposed to produce segment results and rough configuration results at the same time. A measurement unit for the lesion index (LICU) was designed to simplify coarse cluster tests by computing a warm separation chart. For dermoscopic highlight extraction, a straight CNN was suggested. Various injury rates were over 1000 × 700 pixels, requiring high-estimation costs. A deep learning system requires to rescale of injury estimates. Moreover, resizing figures can misrepresent the skin injury. In the first case, a sore figure's middle region has been edited and then comparatively resized to a lower determination. The median area value has been set at 0.8 of the figure height and thus modified with respect to the figure emphasis. Since the exact probability maps of various skin soreness groups provide pathologists with valuable data, the LICU has been suggested to refine the conceived gross skin sore result maps derived from FCRNs.

Dorj et al. [33] proposed a method for skin cancer classification using a deep CNN. The focus of the proposed strategy was the assignment of characterising skin tumours by utilising an ECOC SVM and a profound CNN. A number of figures contained noise such as different organs and apparatuses. These figures were edited to decrease noise for obtaining better results. A current and preprepared AlexNet CNN was utilised for removing highlights. An ECOC SVM classifier was used for skin growth.

Cueva et al. [34] proposed a method for skin cancer detection using computer systems. In their method, figure handling was created to produce the asymmetry, border, color, and diameter of melanoma by utilising neural systems to group various types of moles. Subsequently, this calculation was created after an examination of 200 figures produced an execution of 97.51%. The early identification of skin tumours increases the probability of a cure, such as those found in the cutting-edge stages. In this manner, the death rate of this condition may be reduced. Additionally, late examinations have demonstrated that the estimations of the execution on the arrangement of melanoma by a dermatologist are in the range of 75 to 84%.

Alfed and Khelifi [35] proposed a technique for detecting the types of skin cancers from dermoscopic images. Numerous mechanised methods have been proposed to determine and arrange infections to have agreeable skin disease location execution. Despite this, reducing the false discovery rate is difficult and time consuming because false positives trigger alerts and require mediation by a specialist pathologist for facilitating examination and screening. In this technique, a programmed skin malignancy-finding framework that consolidates diverse textural and shading highlights was proposed. New textural and shading highlights were utilised for effective and exact discovery.

## 3. Preliminaries of Global Optimization

This section provides definitions and assumptions. A general global optimization problem is indicated as follows:

(1) $$\begin{array}{c} \underset{x\in \Lambda }{\min}f\left(x\right), \end{array}$$

where *Λ* ⊂ ℝ^*n*^ is the feasible domain of *x* that is specified by constraints, and *x* = (*x*_1_, ⋯⋯,*x*_*n*_)^*T*^.

Problem (1) is smooth if function *f* is continuously differentiable; otherwise, problem (1) is nonsmooth.

**Definition 1 (see [36]).**

The point *x*^∗^ ∈ *Λ* is said to be a global minimizer of *f* if *f*(*x*^∗^) ≤ *f*(*x*) for all *x* ∈ *Λ*.

**Definition 2 (see [8]).**

The basin, *B*^∗^, of the function, *f*(*x*), at an isolated local minimizer, *x*_*k*_^∗^, is a connected domain containing *x*_*k*_^∗^, in which the steepest descent trajectory of *f*(*x*) converges to *x*_*k*_^∗^ from any initial point in *B*^∗^.

**Definition 3 (see [13]).**

A Bezier curve is characterised by a set of control points, *C*_*n*_, and it is defined as follows:

(2) $$\begin{array}{c} Z\left(t\right)=\overset{n}{\underset{j=0}{\sum }}r_{j,n}\left(t\right)C_{j},0\leq t\leq 1, \end{array}$$

where

(3) $$\begin{array}{c} r_{j,n}\left(t\right)=\left(\begin{array}{c} n\\ j \end{array}\right)t^{j}{\left(1-t\right)}^{n-j}, \end{array}$$

denotes the Bernstein basis polynomials of degree *n*.

The following assumptions are satisfied in the rest of this paper:

*(A1)*. The search should ideally have decent directions; this implies that
  (4) $$\begin{array}{c} d_{k}^{T}\nabla f\left(x_{k}\right)<0. \end{array}$$
*(A2)*. The search directions should be gradient related, so that
  (5) $$\begin{array}{c} \left\|d_{k}\right\|\geq q\left\|\nabla f\left(x_{k}\right)\right\|, \end{array}$$
  where *q* > 0 is a constant.
*(A3)*. The determination of *δ*_*k*_ should include one-dimensional minimisation. This ensures that
  (6) $$\begin{array}{c} f\left(x_{k+1}\right)<f\left(x_{k}\right). \end{array}$$

### 3.1. New Global Optimization Method

The proposed auxiliary function is constructed based on the best local minimizer of *f*(*x*) found so far and the elimination function as

(7) $$\begin{array}{c} \gamma \left(x,x_{k}^{*}\right)=\min\left\{f\left(x\right),f\left(x_{k}^{*}\right)\right\}. \end{array}$$

The typical feature of this function is to remove local minimizers, higher than the previously found minimizer, and keep the original, *f*(*x*), function unchanged in a region in which the function values are lower than the best value of the algorithm. In other words, it has the following properties:

- If *f*(*x*_*k*_^∗^) ≤ *f*(*x*)⟹*γ*(*x*, *x*_*k*_^∗^) = *f*(*x*_*k*_^∗^), for all *x* ∈ *Λ*
- If *f*(*x*_*k*_^∗^) > *f*(*x*)⟹*γ*(*x*, *x*_*k*_^∗^) = *f*(*x*), for all *x* ∈ *Λ*

By utilising multiplication with a piecewise function, *ψ*_*Λ*_1__(*x*), function (7) can be rewritten as

(8) $$\begin{array}{c} \gamma \left(x,x_{k}^{*}\right)=f\left(x_{k}^{*}\right)-\left[f\left(x_{k}^{*}\right)-f\left(x\right)\right]\psi_{\Lambda_{1}}\left(x\right), \end{array}$$

where piecewise function *ψ*_*Λ*_1__(*x*) is defined by

(9) $$\begin{array}{c} \Psi_{\Lambda_{1}}\left(x\right)=\left\{\begin{array}{cc} 1, & x\in \Lambda_{1},\\ 0, & \text{otherwise}, \end{array}\right. \end{array}$$

and includes all possible cases of function *γ*(*x*, *x*_*k*_^∗^) according to the values of *x* and set *Λ*_1_ = {*x* ∈ *Λ* : *f*(*x*_*k*_^∗^) > *f*(*x*)}. All terms of function (8) are smooth except for those related to piecewise function *ψ*_*Λ*_1__(*x*). Hence, it is sufficient to smooth function *ψ*_*Λ*_1__(*x*) to ensure that function (8) is smoothed. By utilising the Bezier curves given by Definition 3, the functions *y*_1_ and *y*_2_ can be defined as follows:

(10) $$\begin{array}{c} y_{1}=\frac{\left(2b_{2}-2b_{1}+2{\left(\left(b_{2}-1\right)\left(b_{1}^{2}\tau -2b_{1}\tau +b_{2}-1\right)\right)}^{1/2}-2b_{1}b_{2}-2b_{1}\tau +b_{1}^{2}b_{2}+b_{1}^{2}\tau -2b_{1}{\left(\left(b_{2}-1\right)\left(b_{1}^{2}\tau -2b_{1}\tau +b_{2}-1\right)\right)}^{1/2}+2\right)}{{\left(b_{1}-2\right)}^{2}},\\ y_{2}=\frac{{\left(b_{1}b_{2}-b_{2}+{\left(b_{2}\left(b_{1}^{2}\tau -2b_{1}\tau +b_{2}\right)\right)}^{1/2}\right)}^{2}}{\left(b_{2}{\left(b_{1}-2\right)}^{2}\right)}, \end{array}$$

where *τ* = *f*(*x*) − *f*(*x*_*k*_^∗^) and *b*_1_ > 0, 0 < *b*_2_ < 1. These functions can be used to obtain the smoothed form of *ψ*_*Λ*_1__(*x*), which can be written as

(11) $$\begin{array}{c} {\tilde{\psi }}_{\Lambda_{1}}\left(\tau ,b_{1},b_{2}\right)=\left\{\begin{array}{cc} 0, & \tau >b_{2},\\ y_{2}, & b_{2}\geq \tau >0,\\ y_{1}, & 0\geq \tau >\frac{-b_{2}}{b_{1}},\\ 1, & \tau \leq \frac{-b_{2}}{b_{1}}. \end{array}\right. \end{array}$$

Thus, the smoothed form of function (8) can be written as follows:

(12) $$\begin{array}{c} \tilde{\gamma }\left(x,x_{k}^{*},b_{1},b_{2}\right)=f\left(x_{k}^{*}\right)-\left[f\left(x_{k}^{*}\right)-f\left(x\right)\right]{\tilde{\psi }}_{\Lambda_{1}}\left(\tau ,b_{1},b_{2}\right). \end{array}$$

**Theorem 1 .**

Suppose *x*_*k*_^∗^ is the local minimizer of *f*, and parameters *b*_1_ and *b*_2_ are defined as above, then we have

(13) $$\begin{array}{c} 0\leq \tilde{\gamma }\left(x,x_{k}^{*},b_{1},b_{2}\right)-\gamma \left(x,x_{k}^{*}\right)\leq \max\left\{b_{2}^{2},\frac{b_{2}-b_{2}^{2}}{b_{1}}\right\}, \end{array}$$

for all *x* ∈ *Λ*.

**Proof**

From the definitions of $\tilde{\gamma }\left(x,x_{k}^{*},b_{1},b_{2}\right)$ and *γ*(*x*, *x*_*k*_^∗^), we have

(14) $$\begin{array}{c} \tilde{\gamma }\left(x,x_{k}^{*},b_{1},b_{2}\right)-\gamma \left(x,x_{k}^{*}\right)=\left(f\left(x\right)-f\left(x_{k}^{*}\right)\right)\left({\tilde{\psi }}_{\Lambda_{1}}\left(\tau ,b_{1},b_{2}\right)-\psi_{\Lambda_{1}}\left(x\right)\right). \end{array}$$

According to the states of *τ* and parameters *b*_1_ and *b*_2_, we consider the following four cases:

**Case 1 .**

If *τ* > *b*_2_, this gives

(15) $$\begin{array}{c} \tilde{\gamma }\left(x,x_{k}^{*},b_{1},b_{2}\right)-\gamma \left(x,x_{k}^{*}\right)=0, \end{array}$$

for *x* ∈ *Λ*.

**Case 2 .**

If *b*_2_ ≥ *τ* > 0, we have

(16) $$\begin{array}{c} \tilde{\gamma }\left(x,x_{k}^{*},b_{1},b_{2}\right)-\gamma \left(x,x_{k}^{*}\right)\leq b_{2}^{2}, \end{array}$$

for *x* ∈ *Λ*.

**Case 3 .**

If 0 ≥ *τ*>−*b*_2_/*b*_1_, we have

(17) $$\begin{array}{c} \tilde{\gamma }\left(x,x_{k}^{*},b_{1},b_{2}\right)-\gamma \left(x,x_{k}^{*}\right)\leq \frac{b_{2}-b_{2}^{2}}{b_{1}}, \end{array}$$

for *x* ∈ *Λ*.

**Case 4 .**

If *τ*≤−*b*_2_/*b*_1_, we have for

(18) $$\begin{array}{c} \tilde{\gamma }\left(x,x_{k}^{*},b_{1},b_{2}\right)-\gamma \left(x,x_{k}^{*}\right)=0, \end{array}$$

for *x* ∈ *Λ*.

As described above, the local removal process loses significant information and contains several removed local minimizers, which are so hard to handle for the algorithm. Improper implementation also leads to additional complications in addressing the global optimization problem. Developing an appropriate method for looking for the best solutions that have been identified so far to find better solutions or basins is important. An escape function, *ζ*, is therefore provided for the treatment of removed local minimizers. This feature is based on the best, *x*_*k*_^∗^, solution that has been found so far, as follows:

(19) $$\begin{array}{c} \tilde{\gamma }\left(x,x_{k}^{*},b_{1},b_{2},a\right)=f\left(x_{k}^{*}\right)-\left[f\left(x_{k}^{*}\right)-f\left(x\right)\right]{\tilde{\psi }}_{\Lambda_{1}}\left(\tau ,b_{1},b_{2}\right)+a\zeta \left({\left\|x-x_{k}^{*}\right\|}^{2}\right), \end{array}$$

where *a* is a real-value constant. *ζ* is an escape function that has the form (1/(1 + ‖*x* − *x*_*k*_^∗^‖^2^)) and satisfies the following properties:

(20) $$\begin{array}{c} \zeta \left(\tau \right)>0,\\ \zeta^{\prime }\left(\tau \right)<0,\\ \lim_{\tau \to \infty }\zeta \left(\tau \right)=0. \end{array}$$

The fundamental properties of auxiliary function (19) can be demonstrated by multiple theorems.

**Theorem 2 .**

Suppose *x*_*k*_^∗^ is a local minimizer of *f* and $\tilde{\gamma }\left(x,x_{k}^{*},b_{1},b_{2},a\right)$ is defined by (19), then point *x*_*k*_^∗^ is a local maximiser of $\tilde{\gamma }\left(x,x_{k}^{*},b_{1},b_{2},a\right)$.

**Proof**

As *x*_*k*_^∗^ is a local minimizer of function *f*, there exists *κ* > 0. *χ* = *N*(*x*_*k*_^∗^, *κ*) is a neighbourhood of *x*_*k*_^∗^, such that *f*(*x*) ≥ *f*(*x*_*k*_^∗^) for any *x* ∈ *χ*. When *x* ≠ *x*_*k*_^∗^, then

(21) $$\begin{array}{c} \frac{\tilde{\gamma }\left(x,x_{k}^{*},b_{1},b_{2},a\right)}{\tilde{\gamma }\left(x_{k}^{*},x_{k}^{*},b_{1},b_{2},a\right)}=\frac{f\left(x_{k}^{*}\right)+\left(a/1+{\left\|x-x_{k}^{*}\right\|}^{2}\right)}{f\left(x_{k}^{*}\right)+a}<1. \end{array}$$

Therefore, we have

(22) $$\begin{array}{c} \tilde{\gamma }\left(x,x_{k}^{*},b_{1},b_{2},a\right)<\tilde{\gamma }\left(x_{k}^{*},x_{k}^{*},b_{1},b_{2},a\right). \end{array}$$

Thus, *x*_*k*_^∗^ is a local maximiser of $\tilde{\gamma }\left(x,x_{k}^{*},b_{1},b_{2},a\right)$.

**Theorem 3 .**

Suppose *x*_*k*_^∗^ is a local minimizer of *f*, then $\tilde{\gamma }\left(x,x_{k}^{*},b_{1},b_{2},a\right)$ has no stationary point for *x* ∈ *Λ*_2_, where *Λ*_2_ = {*x* ∈ *Λ* | *f*(*x*) ≥ *f*(*x*_*k*_^∗^), *x* ≠ *x*_*k*_^∗^}.

**Proof**

In case *τ* = *f*(*x*) − *f*(*x*_*k*_^∗^) > *b*_2_, we have

(23) $$\begin{array}{c} \tilde{\gamma }\left(x,x_{k}^{*},b_{1},b_{2},a\right)=f\left(x_{k}^{*}\right)+a\zeta \left({\left\|x-x_{k}^{*}\right\|}^{2}\right). \end{array}$$

For any *x* satisfying *f*(*x*) ≥ *f*(*x*_*k*_^∗^), we have

(24) $$\begin{array}{c} \nabla \tilde{\gamma }\left(x,x_{k}^{*},b_{1},b_{2},a\right)=a\nabla \zeta \left({\left\|x-x_{k}^{*}\right\|}^{2}\right). \end{array}$$

However, ‖*a*∇*ζ*(‖*x* − *x*_*k*_^∗^‖^2^)‖ > 0 for any *x* ∈ *Λ*_2_, i.e., $\tilde{\gamma }\left(x,x_{k}^{*},b_{1},b_{2},a\right)$ does not have a stationary point at *x* ∈ *Λ*_2_.

**Theorem 4 .**

Suppose *x*_*k*_^∗^ is a local minimizer point of *f* but not global and *f* has a lower minimizer than *x*_*k*_^∗^, then $\tilde{\gamma }\left(x,x^{*},b_{1},b_{2},a\right)$ has a stationary point in *Λ*_1_ = {*x* ∈ *Λ* | *f*(*x*) < *f*(*x*_*k*_^∗^)} if *a* = |*a*| ≤ *L*/*T*, where ‖∇(*aζ*(‖*x* − *x*_*k*_^∗^‖^2^))‖ ≤ |*a*|*T* and ‖∇*f*‖ ≤ *L*.

**Proof**

Selecting parameters *b*_1_ and *b*_2_ to be sufficiently small, our smoothed function, $\tilde{\gamma }\left(x,x^{*},b_{1},b_{2},a\right)$, can be obtained as

(25) $$\begin{array}{c} \tilde{\gamma }\left(x,x^{*},b_{1},b_{2},a\right)=f\left(x\right)+a\zeta \left({\left\|x-x_{k}^{*}\right\|}^{2}\right) \end{array}$$

in the most part of the lower basin. As the norm of the gradient of the function,

(26) $$\begin{array}{c} \zeta \left({\left\|x-x_{k}^{*}\right\|}^{2}\right)=\frac{1}{1+{\left\|x-x_{k}^{*}\right\|}^{2}}, \end{array}$$

is bounded, there exists a number *T* > 0 such that

(27) $$\begin{array}{c} \left\|\nabla \left(a\zeta \left({\left\|x-x_{k}^{*}\right\|}^{2}\right)\right)\right\|\leq \left|a\right|T. \end{array}$$

Hence, the following inequality,

(28) $$\begin{array}{c} \left\|\nabla \left(a\zeta \left({\left\|x-x_{k}^{*}\right\|}^{2}\right)\right)\right\|\leq \left|a\right|T\leq \left\|\nabla f\right\|\leq L, \end{array}$$

enables *f* to increase faster than escape function *ζ* decreases, providing a stationary point in *Λ*_1_, which implies

(29) $$\begin{array}{c} \left|a\right|\leq \frac{L}{T}. \end{array}$$

The idea of the algorithm can be described in the following three important steps:

- The first step is to reduce the objective function into a one-dimensional function in each search direction, *d*_*k*_. The one-dimensional functions are found using *F*_*d*_*k*__(*δ*) = *f*(*x*_0_ + *δd*_*k*_) as a function of *δ*
- The second step is to construct an auxiliary function, $\tilde{\gamma }\left(\delta ,\delta_{k}^{*},b_{1},b_{2},a\right)$, at *δ*_*k*_^*i*^. Point *δ*_*k*_^*i*^ is any arbitrary local minimum of *F*_*d*_*k*__(*δ*), and it is used as an initial point to search for the global minimizer in direction *d*_*k*_
- The third step is to repeat the above phases for all search directions to obtain the local minimizers of *f*(*x*). The lowest among these minimizers is the required global minimizer of *f*(*x*).

## 4. Melanoma Detection Using Global Optimization Algorithm

In this section, the method of global-optimization-based melanoma detection is explained step by step.

**Step 1 .**

The original image is fetched from a database.

**Step 2 .**

The ground truth image is fetched from the database.

**Step 3 .**

In current melanoma skin cancer segmentation, the original grayscale image is preprocessed by employing two transformations. One is the conversion of the grayscale image to RGB, and the other is median filtering conversion. This conversion eliminates hue and saturation but maintains luminance. Median filtering reduces noise such as salt-and-pepper noise.

**Step 4 .**

After median filtering, the histogram of the median image is calculated. It provides information about the intensity distribution of the median image along with the location of the distribution.

**Step 5 .**

The proposed global optimization algorithm is applied to the histogram of the median image using Otsu's method. The weighted sum of the variance of the histogram is considered as a fitness function.

**Step 6 .**

Finally, the global optimization method provides the threshold value for detecting melanoma. This threshold value is compared with the median filtering image. If a point of the image is larger than the threshold value, then the point is changed to white; otherwise, the point is changed to black.

**Step 7 .**

After the image is converted to black and white, an image overlay function is applied to mask the corner of the image. After the masking, the final detected image is generated and compared with the ground truth image.

Sensitivity, specificity, positive predicted value, negative predicted value, accuracy, and computation time are analysed for effective comparison.

The flowchart for global-optimization-based melanoma detection is shown in Figure 1. The steps of global optimization for skin cancer segmentation are shown as a graphical abstract in Figure 2. In this study, for the validation of the proposed optimization process, the PH2 dataset has been used. Every coefficient was evaluated by a competent dermatologist for the numbering factors of analytic performance, the manual partition of lesion areas, and the dermoscopic norm [37].

## 5. Evaluation Results

The International Skin Imaging Collaboration recommends several metrics for performance evaluation. These metrics indicate the performance of each algorithm and method that categorises pixels correctly. Such metrics show the output of each algorithm and process that correctly categorises pixels. This analysis measures precision (Acc (%)), specificity (Spe (%)), positive prediction (PPV), negative predictive value (NPV), and sensitivity (Sen (%)). The following equations are used for the quantitative analysis of the results of all the techniques applied by the various parameters:

(30) $$\begin{array}{c} \text{AC}=\frac{N_{t}p+N_{t}n}{N_{t}p+N_{f}p+N_{t}n+N_{f}n},\\ \text{JA}=\frac{N_{t}p}{N_{t}p+N_{f}n+N_{f}p},\\ \text{DI}=\frac{2\times N_{t}p}{2\times N_{t}p+N_{f}n+N_{f}p},\\ \text{SE}=\frac{N_{t}p}{N_{t}p+N_{f}p},\\ \text{SP}=\frac{N_{t}n}{N_{t}n+N_{f}p}. \end{array}$$

Figure 3 shows the processed melanoma images used to prove the effectiveness of the proposed algorithm. The effectiveness of the proposed method is proved by comparing it with a newly developed method, i.e., the ASLM method^∗^ (details available at 10.1016/j.com-pmedimag.2016.05.002). Six melanoma images are randomly selected, and detection is carried out using the proposed method and ASLM method. The images are shown in Figure 4. The final images obtained by the proposed method are more accurate than those obtained by the ASLM method.  Table 1 shows the comparison of the performance parameters of the global optimization algorithm with JSEG, SRM, KPP, K-means, Otsu, Level Set, and ASLM for 200 image detections. Based on these results, the proposed method produces superior parameters, with a specificity of 0.9928 and an accuracy of 0.9011.

The sensitivity of the proposed method higher than that of the other methods, except the ALSM method. The results obtained using the proposed global optimization method on the PH2 database images of malignant lesions (melanomas) show IMD088 (blue-whitish veil, streaks, and regression areas), IMD284, IMD405, and IMD419 (blue-whitish veil) for the second, third, and fourth rows, IMD424 (blue-whitish veil and streaks) for the fifth row, and IMD425 (blue-whitish veil and regression areas) for the sixth row. The computational speeds for all processing steps are provided in Table 2.

All performance parameters are calculated utilising a stratified cross validation method, in which the PH2 database is divided into three subgroups, each with approximately 40 unhealthy moles and 160 healthy moles for skin cancer lesions.  Table 3 shows a few performance parameters of the six processed images selected randomly from the PH2 database. A recognised statistical assessment parameters are applied to experimentally compare the implementation of the proposed algorithm with existing state-of-the-art segmentation algorithms. The proposed algorithm is applied to 200 benign and melanoma medical images obtained from the PH2 database [38], and the values of the parameters in the algorithm are taken as follows:

(31) $$\begin{array}{c} b_{1}=0.1,b_{2}=0.4,a=1,\varepsilon =0.003,\upsilon =-1,\\ G=100,M=15,ub\left(\text{the upper bound}\right)=10,lb\left(\text{the lower bound}\right)=0. \end{array}$$

From the ISBI 2016 and ISBI 2017 databases, the most complicated images (i.e., images with dermoscopes, bubbles, hair, and multiple colors) have been used in their original dimensions. These databases contain 8-bit dermoscopic RGB images from 540∗722 to 4499∗6748 pixels, with different image dimensions. In addition, both databases included the original images coupled with the boundaries of lesion segmentation, which have been recorded by professional dermatologists.

Figure 5 lists the segmentation results, where the measurement of the comparative methods was taken from the original papers. Deeper learning methods achieve better results than the method in [39], and with the proposed method, the highest Jac and Dic values are obtained. Therefore, the proposed method outperforms comparable methods and segments of skin lesions effectively.

Figure 6 also compares, in terms of Sen, Spe, Acc, Dic, and Jac, the proposed approach and other common methods employed by the ISBI 2017 database.

According to uneven skin patches, such as freckles, dermoscopic image repositories could have several small objects.

Such small objects can be screened out by using the median filter. In some cases, all impurities are not removed and the filter has an impact on algorithm work and results.

Figure 7 shows images that fail to the segment. The color contrast of skin lesion and underlying skin in rows 2 and 3 is identical. In this case, the optimal threshold value is difficult to determine because of color differences between the skin lesions and the background with no noticeable pigmentation in the lesions. If the contrast between the skin lesion and the skin around is not sufficient enough, the gray threshold algorithm of global optimization takes in a large part of the skin around the image and stretches to the edge of the image. It also causes a segmentation failure as the mask reaches the image's edge. Considering that the primary skin lesion is an adjacent area, segmented images should first involve only one adjacent context with no isolated elements or troughs. The first area (including the image) can be of any size and possibly bordering the image. This is why the image failed in row 1.

The comparison of state-of-the-art methods and the global optimization algorithm is provided in Table 4. If sensitivity is considered as the most significant component, which implies that every patient with skin cancer is detected, the global optimization algorithm has the highest performance. Thus, the global optimization algorithm is suitable for finding and segmenting melanoma skin cancer.

## 6. Conclusion

In this paper, a new method is proposed for melanoma skin cancer segmentation. The method is based on the global optimization technique, and it uses an auxiliary function for performing directional search via Bezier curves. The proposed algorithm is a fully automatic detection technique that does not require a training phase. Moreover, its computation time for detecting melanoma images is extremely short. The proposed method is verified experimentally using three public dermoscopic image databases. The performance of the proposed algorithm is compared with the existing melanoma segmentation techniques in terms of sensitivity, specificity, and accuracy. Evaluation test results show that our proposed segmentation method outperforms the other conventional state-of-the-art segmentation algorithms, and its efficiency is comparable to the new approaches based on deep neural networks. The proposed method is suitable for melanoma segmentation in skin cancer diagnosis.

## Figures and Tables

**Figure 1:** Flowchart for the segmentation process using the proposed global optimization method.

**Figure 2:** Steps of global optimization method for skin cancer segmentation.

**Figure 3:** Ten sets of images for melanoma detection using global optimization algorithm.

**Figure 4:** Comparison of proposed method and ASLM method.

**Figure 5:** Comparison of earlier studies with the current method for ISBI 2016 database [2, 4, 40–42].

**Figure 6:** Comparison of earlier studies with the current method for ISBI 2017 database [32, 38, 43–48].

**Figure 7:** A variety of segmentation failure cases: Row (1-3) PH2, ISBI 2016, and ISBI 2017 datasets; Columns (a) original image; (b) manual segmentation image (ground truth); (c) proposed method segmentation image; and (d) result of proposed method (green) and ground truth (red).

**Algorithm 1:** Algorithm

**Table 1:** Performance parameter results for 200 image detections from the PH2 database.

Method	Sen	Spe	Acc
Otsu (MATLAB 2014a)	0.5221	0.7064	0.6518
SRM [49]	0.6518	08757	0.6766
KPP (MATLAB 2014a)	0.4147	0.9581	0.7815
Level set [50]	0.7188	0.8003	0.7842
K-means (open CV2.4)	0.7291	0.8430	0.8249
JSEG [51]	0.7108	0.9714	0.8947
ASLM	0.8024	0.9722	0.8966
Global optimization algorithm	0.8892	0.9933	0.932

**Table 2:** Total time consumed by the proposed method for six images selected randomly from 200 images in the PH2 database.

Proposed method (global optimization)	Total time consuming (sec)
Image processing	19.25 ± 2.02
Classification	(18.27 ± 12.13) × 10^−3^

**Table 3:** Comparison of performance parameters for the five processed images selected randomly from the PH2 database.

Image no.	PPV	NPV	Computation time (sec)
1	0.901184	0.999942	3.312
2	1	0.988564	3.407
3	0.984021	1	3.489
4	0.970134	0.997304	3.579
5	0.924157	0.998954	3.357
6	0.9327	0.9898	3.217

**Table 4:** Comparison of the proposed algorithm with state-of-the-art methods.

		Number of cases			
References	Benign	Melanoma	Sen (%)	Spe (%)	Acc (%)
D'Amico and Stanganelli [52]	927	50	96.41	87.16	91.78
Tanaka et al. [53]	181	70	90.00	98.30	94.00
Maglogiannis and Kosmopoulosb [54]	14	20	90.00	93	94.00
Marques et al. [55]	146	17	94.10	77.40	85.50
Olszewska and Semantic [56]	24	24	100	66.66	83.33
Zagrouba and Barhoumi [57]	160	40	71.30	93.50	82.00
Aljanabi et al. [58]	160	40	95.50	98.40	96.02
Proposed global optimization algorithm	160	40	95.93	98.99	96.28

## Data Availability

The PH2 database means the Pedro Hispano Hospital that deals with dermatology by dermoscopic images in a Tubingen Mole Analyzer system. This data set is free and open source and all people they can use these data set. Also we used these data set to our proposed method.
